RETRACTED

# Optimizing sowing date for peanut genotypes in arid and semi-arid subtropical regions

**DOI:** 10.1371/journal.pone.0252393

**Published:** 2021-06-10

**Authors:** Muhammad Ijaz, Ahmad Nawaz, Sami Ul-Allah, Ahmad Sher, Abdul Sattar, Muhammad Sarwar, Ijaz Hussain, Anees Ur Rehman, Muhammad Ashfaq Wahid, Mohammad Javed Ansari, Kamel Hessini

**Affiliations:** 1 College of Agriculture, Bahauddin Zakariya University, Bahadur Sub-Campus Layyah, Pakistan; 2 Center for Agriculture and Biosciences International (CABI), Central and West Asia (CWA), Satellite Town Rawalpindi, Pakistan; 3 Agricultural Extension & Adaptive Research Department, Government of the Punjab, Lahore, Pakistan; 4 Department of Agronomy, University of Agriculture, Faisalabad, Pakistan; 5 Department of Botany, Hindu College Moradabad (Mahatma Jyotiba Phule Rohilkhand University Bareilly), Moradabad, India; 6 Department of Biology, College of Sciences, Taif University, Taif, Saudi Arabia; Harran Üniversitesi: Harran Universitesi, TURKEY

## Abstract

Peanut (*Arachis hypogea* L.) is an important nut crop extensively grown in rainfed regions of Pakistan. The crop requires low inputs; thus, could grow successfully under diverse environmental conditions. Due to pegging ability, peanut grows aggressively in sandy and sandy-loam soils. However, it has not introduced to Thal region of southern Punjab, Pakistan. A two-year field experiment was conducted to optimize sowing dates for two peanut genotypes (‘BARI-2016’ and ‘NO-334’) in Thal region (Layyah). Similarly, a yield trial was conducted at Chakwal where both genotypes are extensively grown. Five sowing dates (10^th^ April, 1^st^ May, 20^th^ May, 10^th^ June and 30^th^ June) were included in the study. The highest seed yield was obtained with early sown crop (10^th^ April) during both years. Pod formation reduced with increasing atmospheric temperature and no pods were formed on the plants sown on 30^th^ June. Decreased pod formation seemed a major reason for low yield in late-sown crop. The highest yield was observed for the crop sown on 10^th^ April, which was decreased by 40% for the crop sown on 1^st^ May. Genotype ‘BARI-2016’ performed better for seed yield at both locations compared with ‘NO-334’. The results suggested that genotype ‘BARI-2016’ is more adaptive to arid and semi-arid condition under rainfed or irrigated conditions. Sowing peanut at optimum time would increase seed yield in arid and semi-arid regions. Nonetheless, ‘BARI-2016’ can be grown under rainfed and irrigated conditions successfully.

## Introduction

Peanut (*Arachis hypogaea* L.) is a self- pollinated, annual, leguminous oilseed and nut crop that can fix atmospheric nitrogen [1]. It is mostly grown in arid and semi-arid regions of the world with warm to equatorial climates [2, 3]. Although peanut can tolerate wide range of pH, its better growth and development is observed under neutral pH and on marginally acidic soils [4]. The atmospheric/soil temperatures >45 °C and <15 °C impede seed germination of peanut [5]. Extremely low temperatures during early or late crop developmental stages may result in immature pods, while high temperatures are responsible for retarded crop growth rate and moisture stress [6–9].

RETRACTED

Peanut is adapted to a wide range of soil types and environments; however, yield is highly sensitive to environmental conditions [10, 11]. Furthermore planting significantly affects yield and quality attributes of peanut [12, 13]. Sunlight and temperature have greater effects on the productivity of peanut as both are directly involved in several phenological phenomenon. It is reported that peanut can be successfully grown under a wide range of sowing times; however, early or late planting significantly affects yield depending on the region [14]. Likewise, selection of a suitable cultivar is also associated with planting time as early or late sown genotypes are available for almost all crops. Fluctuating temperatures due to varied planting dates significantly influence growth and productivity of peanut [6, 15].

There is a large gap between consumption and domestic production of edible oil in Pakistan. Unfortunately, cultivation of oilseed crops is confined to a limited area (except cottonseed) due to their low yield. Peanut is cultivated mainly in rainfed areas of Punjab (84%), Khyber Pakhtunkhwa (13%) and Sindh (3%) provinces of Pakistan [16]. There are many other potential areas that could be used to increase the national production of peanut. Thal region is one of the potential area, which is arid to semi-arid with subtropical climate. However, the region receives low rainfall (~250 mm per annum), and supplementary irrigation could be used to overcome moisture deficiency. There is a dire need to explore the region for introduction of peanut.

Keeping in view the facts described above, a comprehensive experiment was planned to optimize planting time for two peanut cultivars in semi-arid subtropical regions (Thal) with supplemental irrigation. Comparing yields of the genotypes Chakwal (hub for peanut production in Pakistan) and Layyah (Thal region) was the second major objective of the study.

## Materials and methods

### Experimental site and treatments

A two-year Field experiment was conducted at experimental farm of College of Agriculture, Bahauddin Zakariya University, Sub-campus Layyah (longitude 70° 58’, latitude 31° 01’ and 147 meters asl). Since precipitation do not fulfill the water requirements, supplemental irrigation was applied to exclude the effects of moisture stress. The experiment was repeated (for yield data only) under rainfed conditions in Chakwal (longitude 72° 52’, latitude 32° 56’ and 524 meters asl). Chakwal is rainfed, major peanut production hub with subtropical semi-arid climate, whereas Layyah has similar climate but supplemental irrigations are necessary due to low rainfall. Weather data of both experimental locations for crop duration are given in S1 Table.

RETRACTED

Seeds of ‘BARI-2016’ and ‘NO-334’ genotypes were obtained from Barani Agriculture Research Institute, Chakwal, Punjab, Pakistan. The ‘BARI-2016’ is newly approved peanut genotype for general cultivation. It is bunch type (erect) having high yield potential with moderate tolerance to biotic and abiotic stresses. The ‘NO-334’ is an old and spreading genotype, which has been under cultivation due to good yield potential. On the other hand, it has very low tolerance to biotic and abiotic stresses.

Experimental treatments include five sowing dates (10^th^ April, 1^st^ May, 20^th^ May, 10^th^ June and 30^th^ June) and two peanut genotypes (‘BARI-2016’ and ‘NO-334’). The experiment was laid out according to randomized complete block design with split-plot arrangements where sowing dates were kept in main plots, while genotypes were placed in sub-plots.

### Soil properties

Soil samples were collected from both locations before the cultivation of the crop. At both locations, experimental plots were fallow before the initiation of experiments during both years. Averaged over two years, soil of Layyah was sandy-loam with 8.0 pH, 3.42 dS m^-1^ electrical conductivity, 0.59% organic matter, 600 mg kg^-1^ nitrogen, 137 mg kg^-1^ potassium and 7.5 mg kg^-1^ phosphorus. Experimental soil at Chakwal was sandy-loam with 7.4 pH, 1.13 dSm^-1^ electrical conductivity, 0.45% organic matter, 390 mg kg^-1^ nitrogen, 87 mg kg^-1^ potassium and 5.7 mg kg^-1^ phosphorous.

### Crop husbandry

The row-to-row distance for ‘BARI-2016 and NO-334’ was kept 40 and 50 cm, respectively, while plant-to-plant spacing was 20 cm. Seeds were sown in lines (one seed per hill) with the help of a dibbler. Seeds were dibbled by maintaining seeding depth of 7 cm. Experiment consisted of 30 experimental units (5 sowing date × 2 genotypes × 3 replications) at each site with a net plot size of 2.4 m × 4 m for ‘BARI-2016’ and 3 m × 4 m for ‘NO-334’.

No irrigation was applied at Chakwal as crop relied on monsoon precipitation. Under irrigated conditions at Layyah, pre-sowing irrigation was applied and subsequent irrigations were applied keeping in view crop water requirements, critical growth stages and prevailing weather conditions. A total 8 irrigations of 75 mm each were applied at Layyah during each growing season. Recommended doses of nitrogen, potassium and phosphorus were applied at both locations. The crop sown at first two sowing dates was harvested during the first fortnight of November, while crop sown on other three sowing dates was harvested in the second fortnight of November at both sites.

RETRACTED

### Data collection

Number of leaves per plant, root dry weight and number of nodules were recorded for the crop sown at Layyah during both years. Three plants were harvested from each plot at 30, 60 and 90 days after sowing, and the numbers of leaves and nodules per plant were counted and averaged. The roots of same plants were separated and dried in an oven until constant dry weight to record root dry weight.

Increase in number of leaves per plant per day was calculated by following formula

$$Number\;of\;leaves\;per\;day=\frac{L_{2}-L_{1}}{number\;of\;days}$$

Here, L_1_ is number of leaves at 1^st^ harvest and L_2_ is number of leaves at last harvest.

Formation of nodules per day was calculated by following formula

$$Number\;of\;Nodules\;per\;day=\frac{N_{2}-N_{1}}{number\;of\;days}$$

Here, N_1_ is number of nodules at 1^st^ harvest date and N_2_ is number of nodules at last harvest.

Accumulation of root biomass per day was calculated by following formula

$$Accumulation\;of\;root\;dry\;biomass=\frac{{DM}_{2}-{DM}_{1}}{number\;of\;days}$$

Here DM_1_ is root dry biomass at 1^st^ harvest and DM_2_ is root dry biomass at last harvest.

Data relating to number of pods (one, two, three seeded and total) and seed yield were recorded for both sites. Two central rows from each plot were harvested at maturity with the help of a digger and one, two and three seeded pods were counted, separately and averaged. All types of pods (except empty pods) were calculated and averaged. The separated pods were sun dried (up to 10% moisture contents) and shelled to calculate seed yield.

### Statistical analysis

Due to differences in climate data for the locations were analyzed separately. Data relating to number of leaves, number of nodules and root dry biomass were presented in the form of line graph with periodic data. Data for yield and related traits were s analyzed by two-way analysis of variance (ANOVA). Tukey’s post-hoc test was used to separate the means where ANOVA denoted significant differences (p≤0.05).

## Results

### Phenological data

The number of leaves and nodules per plant and root dry weight increased with time. The number of leaves were nearly same for all sowing dates at 30 days after sowing (DAS) in both genotypes, except for 30^th^ June sowing where leaves were less. Higher number of leaves were produced by genotypes ‘NO-334’ than ‘BARI-2016’. The highest number of leaves were observed for 10^th^ April and 1^st^ May sowing on genotype ‘BARI-2016’ at 90 DAS, while ‘NO-334’ produced higher number of leaves for 10^th^ April sowing (Fig 1A). For increase in number of leaves per day, differences were minimum until 60 DAS for both genotype and sowing dates; however, at 90 DAS, the rate of leaf formation was higher for 20^th^ April and 1^st^ May sowing in genotype ‘BARI-2016’. Overall, rate of leaf formation was higher in genotype ‘NO-334’ than ‘BARI-2016’ (Fig 1B).

RETRACTED

**Fig 1:** Effect of sowing date and genotype on A) number of leaves per plant and B) increase in number of leaves per plant per day. Each value is average of two years and three replications (n = 6).

Interestingly, 30 DAS, number of nodules per plant in both genotypes were higher for 10^th^ June sowing. However, early sowing recorded higher number of nodules at 60 DAS. Similarly, crop sown on 1^st^ April recorded the highest number of nodules at 90 DAS and genotype ‘BARI-2016’ had higher number of nodules than ‘NO-334’ (Fig 2A). Regarding nodule formation rate, sowing dates had little differences until 30 DAS. Nodule formation rate increased for first three sowing dates, while decreased for 10^th^ June sowing at 30–60 DAS. A fast increase was observed for the crop sown on 1^st^ April and genotype ‘BARI-2016’ recorded higher nodule formation rate than ‘NO-334’ (Fig 2B).

**Fig 2:** Effect of sowing date and genotype on A) number of nodules per plant and B) increase in number of nodules per plant per day. Each value is average of two years and three replications (n = 6).

Root dry biomass increased for both genotype and all sowing dates until 90 DAS and a decreasing trend was recorded in root biomass with delayed sowing. Genotype ‘BARI-2016’ recorded similar pattern of root dry biomass for all sowing dates until 60 DAS. However, genotype ‘NO-334’ observed no difference in root biomass for 1^st^ May, 20^th^ May and 10^th^ June sowing with the highest root dry biomass observed for 20^th^ April sowing (Fig 3A). Dry root biomass accumulation rate decreased for first three sowing dates from 30–60 DAS, but remained nearly same for 10^th^ and 30^th^ June sowing. For both genotypes dry root biomass accumulation rate was higher for 20^th^ April sowing. Dry root biomass accumulation rate increased for all sowing dates in ‘BARI-2016’ (Fig 3B).

**Fig 3:** Effect of sowing date and genotype on A) root dry biomass (g) per plant and B) increase in root dry biomass (g) per plant per day. Each value is average of two years and three replications (n = 6).

RETRACTED

#### Yield components and yield

Analysis of variance indicated that sowing dates and genotypes differed significantly (p≤0.05) for one seeded, two seeded and three seeded pods per plant. Although plants were germinated and grown up for 30^th^ June sowing, no pod was formed during 2017 whereas little pod formation was noted during 2018. Sowing date by genotype interaction was significant (p<0.05); therefore, means were compared across genotypes and sowing dates.

The highest values of single and double seeded pods were recorded for genotype ‘NO-334’ with 10^th^ April sowing. Likewise, the highest values of three seeded pods were observed for ‘BARI-2016’ during both years (Table 1). Genotype ‘BARI-2016’ performed better for three seeded pods during both years. The maximum number of pods (total) was observed for ‘NO-334’ during both years with 10^th^ April sowing. Higher values for total number of pods were observed during 2017 (51 pods per plant) than 2018 (44 pods per plant). The lowest number of all types of pods were recorded for the crop sown on 30^th^ June (Table 1).

**Table 1:** Influence of sowing date and genotype on one, two and three seeded pods per plant under semi-arid subtropical climates (Layyah).

Sowing Dates	2017			2018		
	BARI-2016	NO-334	Mean (G)	BARI-2016	NO-334	Mean (G)
**One seeded pods per plant**						
10-April	12.4 bc	23.9 a	18.2 A	15.4 b	20.2 a	17.8 A
01-May	12.9 bc	15.7 b	14.3 AB	13.7 b	15.2 b	14.5 B
20-May	14.9 bc	7.5 cd	11.2 B	13.1 b	10.7 c	11.9 C
10-June	2.93 d	2.93 d	2.93 C	6.1 d	8.2 cd	7.2 D
30-June	0.00	0.00	0.00	2.2 e	2.3 e	2.3 E
**Mean (SD)**	10.8	12.5		10.1	11.3	
**Two seeded pods per plant**						
10-April	14.8 bc	26.8 a	20.8 A	16.4 b	22.0 a	19.2 A
01-May	13.8 bc	16.0 bc	14.9 B	13.2 bc	15.2 b	14.2 B
20-May	20.1 ab	11.3 cd	15.7 B	10.1 c	12.5 bc	11.3 C
10-June	2.93 d	3.20 d	3.07 C	6.9 d	5.1d e	6.0 D
30-June	0	0	0	2.5 e	2.8 e	2.7 E
**Mean (SD)**	12.9	14.4		9.8	11.5	
**Three seeded pods per plant**						
10-April	3.97 a	0.47 e	2.22 A	3.70 a	1.83 bc	2.77 A
01-May	2.43 b	0.50 e	1.47 AB	2.23 b	0.77 c	1.50 B
20-May	1.90 c	0.35 e	1.13 B	1.33 c	1.03 c	1.18 C
10-June	1.00d	0.20 e	0.60 B	1.10 c	0.43 d	0.77 DE
30-June	0	0	0	0.67 d	0.5 d	0.59 E
**Mean (SD)**	2.3 A	0.4 B		1.81 A	0.91 B	
**Number of pods per plant**						
10-April	33.1 bc	51.2 a	42.2 A	35.5 b	44.0 a	39.8 A
01-May	29.2 bc	32.2 bc	30.7 B	29.1 bc	31.2 bc	30.2 B
20-May	36.4 b	19.0 cd	27.7 B	24.5 c	24.2 c	24.4 C
10-June	6.53 d	6.20 d	6.37 C	14.1 d	13.8 d	13.9 D
30-June	0.00	0.00	0.00	5.4 e	5.6 e	5.5 E
Mean (SD)	26.3	27.2		21.7	23.8	

SD = sowing dates; G = peanut Genotypes

For interaction (sowing date ×genotypes) lettering is done across two columns in each year. Values sharing same letter in each year does not have any significant (p>0.05) difference

The highest yield was observed at Layyah for 10^th^ April sowing during both years. However, yield was nearly double for 1^st^ May and 20^th^ May sowing at Chakwal compared to Layyah. Yield was comparable for 10^th^ and 20^th^ June sowing. It should be mentioned here germination occurred for 30^th^ June sowing during 2017 but no pods were formed; therefore, yield is mentioned zero. Likewise, due to dry period crop could not be grown on 10^th^ June at Chakwal; therefore, yield is mentioned as zero (Table 2).

RETRACTED

**Table 2:** Influence of sowing date and genotype on seed yield (tons/ha) of peanut grown under semi-arid subtropical climates (Layyah) and rainfed arid subtropical climate (Chakwal).

	Layyah						Chakwal					
	2017			2018			2017			2018		
	BARI-2016	NO-334	Mean (G)	BARI-2016	NO-334	Mean (G)	BARI-2016	NO-334	Mean (G)	BARI-2016	NO-334	Mean (G)
10-April	1.06 b	1.23 a	1.15 A	0.96 b	1.20 a	1.08 A	1.12 a	0.85 b	0.98 A	1.00 a	0.81 b	0.91 A
01-May	0.67 c	0.72 c	0.69 B	0.70 c	0.55 cd	0.63 B	1.10 a	0.80 bc	0.95 A	0.90 ab	0.65 c	0.78 B
20-May	0.45 d	0.27 de	0.36 C	0.51 cd	0.32 d	0.42 C	0.93 b	0.71 c	0.82 A	0.75 b	0.54 cd	0.65 B
10-June	0.46 e	0.34 e	0.40 C	0.41 d	0.30 e	0.36 CD	0.00	0.00	0.00	0.40 d	0.30 d	0.35 C
30-June	0.00	0.00	0.00	0.30 e	0.20 f	0.25 D	0.50 d	0.34 d	0.42 B	0.21 e	0.15 e	0.18 D
Mean (SD)	0.70	0.60		0.62 A	0.47 B		0.91A	0.67 B		0.65 A	0.49 B	

SD = sowing dates; G = peanut Genotypes

For interaction (sowing date ×genotypes) lettering is done across two columns in each year. Values sharing same letter in each year does not have any significant (p>0.05) difference

## Discussion

Genotype and sowing dates are two most important attributes for successful production of any crop in a specific agro-ecological zone. In the current study, performance of two peanut genotypes was evaluated at two locations. For both genotypes, 30^th^ June sowing was unsuitable, no pods were formed during 1^st^ year and the lowest yield was recorded for this sowing date during 2^nd^ year. The lowest yield of 30^th^ June sowing is attributed to unfavorable day length and climatic conditions, resulting in low pods setting [17–19]. Kelly et al. [19] reported that extended photoperiod increases vegetative growth and decreases reproductive growth, which result in lesser pod formation and ultimately lower yield. Increase in number of leaves reflects increased vegetative growth. This increase was relatively slow till 60 DAS for all sowing dates due to parallel reproductive growth [18, 19]. However, number of leaves increased rapidly for early sowing, but remained slow for late sown crop due to unfavorable environmental conditions, slow reproductive growth [19] and lower light use efficiency [15]. Nodule formation rate increased during 60–90 DAS, especially for early sowing, which is attributed to more rainfall and humidity during July and August resulting in moderate temperature and high microbial activities in the soil [20, 21]. Abd-Alla et al. [21] reported that harsh soil environment is detrimental for root nodule formation in legumes leading to lower number of nodules and lower efficiency of N-fixing bacteria. Genotypic differences existed due to presence of different genes controlling the specific traits [22, 23] and the expression pattern of transcription factors also vary between the genotypes [24].

RETRACTED

Number of pods (one, two, three seeded and total) were similar for first three sowing dates, but remained very low for June sowing. It shows June sowing is not feasible in Layyah due to high temperature during early flowering and pod formation [25, 26]. Dhanaraj [25] reported that temperature >36 °C severely affects pollen viability of peanut leading to less pod and seed formation. Likewise, Gulluoglu et al. [26] showed negative impact of high temperature on reproductive growth and yield of peanut. Therefore, in current study, lower pod formation is attributed to poor reproductive growth of late-sown peanut leading to poor pod development and lower yield. For the first sowing date, genotype ‘NO-334’ produced higher number of pods and better yield during both years.

Genotype ‘BARI-2016’ performed better than ‘NO-334’ at both locations, which is attributed to its better adaptability under diverse environmental conditions. Looking at the yield, sowing of peanut on 10^th^ April is more productive for both genotypes at Layyah. However, at Chakwal, 10^th^ April and 1^st^ May sowing were statistically at par. Differences in the performance of genotypes at different location is attributed to genotype and environment interaction as reported earlier [22, 27].

## Conclusion

Sowing date and genotype matter for peanut adaptation to any agro-ecological region. Yield of peanut decreased by 40% in both genotypes with delayed sowing by 20 days. Earlier sowing than 10^th^ April in Layyah location is not feasible due to pre-planted chickpea and wheat crops. For Chakwal, both 10^th^ April and 1^st^ May were statistically at par. Genotype ‘BARI-2016’ remained more adaptive to Layyah and Chakwal locations than ‘NO-334’. Therefore, it is recommended that peanut must be sown from 10^th^ April to 1^st^ May for higher yield and economic returns.

RETRACTED

## Supporting information

S1 Table Weather data during the both experimental year at Chakwal and Layyah site. (DOCX)
